# The role of chromium supplementation in cardiovascular risk factors: A comprehensive reviews of putative molecular mechanisms

**DOI:** 10.1016/j.heliyon.2023.e19826

**Published:** 2023-09-04

**Authors:** Dhiaa lattef Gossa Al-Saadde, Ali Murtaza Haider, Arsalan Ali, Ebraheem Abdu Musad Saleh, Abduladheem Turki Jalil, Furqan M. Abdulelah, Rosario Mireya Romero-Parra, Nahla A. Tayyib, Andrés Alexis Ramírez-Coronel, Ameer S. Alkhayyat

**Affiliations:** a Department of Internal Medicine, College of Medicine, Basrah University Teaching Hospital, Basrah, Iraq; b Faisalabad Medical University, Faisalabad, Pakistan; c Rawalpindi Medical University, Rawalpindi, Pakistan; d Department of Chemistry, Prince Sattam Bin Abdulaziz University, College of Arts and Science, Wadi Al-Dawasir, 11991, Saudi Arabia; e Medical Laboratories Techniques Department, Al-Mustaqbal University College, Babylon, Hilla, 51001, Iraq; f College of Pharmacy, Al-Bayan University, Baghdad, Iraq; g Department of General Studies, Universidad Continental, Lima, Peru; h Faculty of Nursing, Umm Al-Qura University, Makkah, Saudi Arabia; i Catholic University of Cuenca, Azogues Campus, Ecuador; j University of Palermo, Buenos Aires, Argentina; k National University of Education, Azogues, Ecuador; l CES University, Colombia; m Medical Laboratory Technology Department, College of Medical Technology, The Islamic University, Najaf, Iraq

**Keywords:** Cardiovascular diseases, Chromium, Hypertension, Inflammation, Oxidative stress

## Abstract

In the recent years, micronutrients play an important role in improving body health with preventing and treating of chronic diseases. Chromium is one of the vital minerals involved in the regulation of insulin action. According to abundant evidences this mineral seems to be an essential factor involved in the reduction of insulin resistance and decreasing the risk of type 2 diabetes mellitus (T2DM) and cardiovascular diseases (CVDs). Moreover, it has been proposed that Chromium supplementation affects mechanisms involved in blood pressure, lipid metabolism, inflammation, and oxidative stress. For instance, it may affect blood pressure through alteration of the renin-angiotensin system, as well as reducing the angiotensin-converting enzyme activity. Furthermore, Chromium supplementation might help *reduce the* coronary *heart disease rates*. This study aims to provide a comprehensive review regarding to the effects of Chromium supplementation on CVDs risk factors with an emphasis on possible molecular mechanisms.

## 1 Introduction

The cardiovascular system includes a large part of the body including the heart, blood vessels, and almost 5 L of blood. A large variety of health problems are associated with the cardiovascular system such as rheumatic heart disease, endocarditis, and conduction system abnormalities [1]. According to recent reports, CVDs have been considered as one of the two contributing causes of mortality and morbidity in the United States since 1975 with 633,842 death numbers or 1 in every 4 deaths [2]. CVD has been considered the major reason of mortality in 2015 followed by 595,930 cancer-related death [2]. Based on World Health Organization (WHO) assessment in 2015, CVDs are the leading cause of worldwide death, taking an estimated 17.7 million lives each year. Of note, CVD has been considered one of the costly diseases even ahead of diseases like Alzheimer and diabetes. Scientists proportionated the indirect costs of $237 billion dollars to CVDs in a year and then expected to reach $368 billion till 2035 [1,3].

There is a close relationship between CVDs and T2DM, this association is more highlighted in heart failure (HF), ischemic heart disease, coronary artery disease (CAD), stroke, and peripheral artery diseases, which these complications are the main causes of death for at least 50% of patients with T2DM [4,5]. In addition, insulin resistance and elevated blood sugar leads to macro and micro-vascular complication in T2DM patients. Besides, abnormal lipid profiles contributes to insulin resistance, fibrosis, and diastolic dysfunction [4]. Of note, CVDs refers to the following four entities: peripheral artery disease (PAD), coronary heart disease (CHD), cerebrovascular disease, and aortic atherosclerosis [1]. Atherosclerosis is the most common entity of CVDs [6]. It is the pathogenic process in the arteries and the aorta that can potentially contribute to a consequence of decreased or absent blood flow from stenosis of the blood vessels [7]. Previous investigations showed that the pathophysiological nature of atherosclerosis initiates endothelial dysfunction [7]. The stimulating factors for atherosclerosis include hypercholesterolemia, hypertension, smoking, hyper-homocysteinemia, impaired glucose metabolism, and infections [1]. In particular, the factors involved in impairing endothelial function such as serum elevated levels of low-density lipoproteins (LDL), and also oxidative stress play key roles in atherosclerosis pathophysiology [8].

CVDs were previously treated by medications and lifestyle modifications. However, the application of these treatments was often fruitless and poor. The emergence of complementary therapies appears to be a vital method for physicians to be aware of the risks and advantages of these options [[9], [10], [11], [12]]. Amongst various treatment strategies, the use of natural products and minerals seems to be safe, efficient and found naturally in foods [[13], [14], [15], [16], [17]]. It has been shown that minerals such as selenium, magnesium, calcium and chromium can play an important role in cardiovascular health [13,[18], [19], [20]]. For instance, chromium is a vital mineral that plays a crucial role in regulating the insulin function, metabolic syndrome, and CVDs [21,22]. According to the results of recent studies, trivalent chromium acts as a cofactor in the activation of insulin as a hormone that mediates the metabolism of lipids, proteins and carbohydrates, and thus can play a role in the prevention and treatment of T2DM and CVDs [23]. It has been revealed that the levels of plasma Chromium in patients with CVDs are considerably lower than in normal subjects [22]. Therefore, Chromium supplementation can be considered as a promising treatment for CVDs [24]. Besides, Chromium can facilitate insulin signaling; it may affect and improve systemic insulin sensitivity [21]. In a recent study, the effects of chromium supplementation (commonly used picolinate or novel form as nanoparticles) and switching away from obesogenic dietary habits on the parameters of lipid metabolism, inflammation, and oxidative stress in liver and plasma of obese rats, has been investigated and the results showed that this supplement can reduce inflammation and oxidative stress as well as improve lipid metabolism [25]. Also, several studies have shown the Chromium supplementation role in carbohydrate and lipid metabolism [26], blood pressure changes [27], the level of oxidative stress markers [28], inflammatory indices [13], liver enzymes, and body mass index (BMI) [29].

Although Chromium supplementation seems to be a safe treatment for control of CVDs risk factors and its deficiency is a major risk factor for this condition, epidemiological data on Chromium intake and involved mechanisms are still limited. Hence, the aim of this study is to reveal the possible protective role of Chromium against CVDs and the possible related mechanisms.

### 1.1 Chromium effects on blood pressure

It has been shown that Chromium supplementation can play a role in the prevention and treatment of CVDs [30]. It has been evidenced that individuals suffered from CVDs have shown lower plasma Chromium levels compared to healthy subjects [22,31]. Epidemiological studies suggested that the use of Chromium and its plasma levels may play a key role in regulating blood pressure [27,32,33]. This supplement improves blood pressure in diabetic patients with hypertension [29]. It has been shown that a higher dose of Chromium can improve blood pressure by decreasing diastolic blood pressure (DBP) [34]. Furthermore, the higher Chromium dose appears to be associated with a better response to systolic blood pressure (*SBP*) [29].

A number of studies reported that the Chromium intakes at dose of 400 and 42 μg (in combination with 9 g brewer's yeast) during 12 and 4 weeks have been related to SBP reduction [35,36]. Moreover, in a study, individuals with systolic dysfunction have been shown with higher serum Chromium levels compared to those with normal systolic function [37]. A systematic reviews and meta-analyses also indicated that Chromium supplementation may have protective effects against myocardial infarction, reduce CVD-associated inflammatory biomarkers [13], and decrease DBP [34]. Conversely, in one study, the negative correlation between plasma Chromium levels and blood pressure and low-density lipoproteins has been reported [27]. A number of studies have presented that Chromium supplementation has no effect on SBP or DBP [[38], [39], [40], [41], [42], [43], [44], [45], [46]]. In the study that conducted by Nussbaumerov et al., in 2018, chromium supplementation at a dose of 300 μg/day for 24 weeks had no effect on blood pressure levels in patients with T2DM [40]. Similarly, a study which was performed by Kalbasi et al., in 2014, with a dose of 200 μg Chromium-enriched during 12 weeks, had no effects on SBP and DBP in T2DM patients [41] (Table 1).

**Table 1:** Effects of chromium supplementation on blood pressure and lipid profile indices in clinical trial studies.

Author (year)	Country (Reference number)	Study design (Sex) Heath Situation	Participants numbers (Intervention/Placebo)	Dose of chromium Administered/day (Mean age)	Duration	Outcome measures
Yanni et al. (2018)	Greece [35]	Parallel (M/F) T2DM patients	30 (15/15)	400 μg chromium- enriched yeast bread (65.8 years)	12 weeks	↓ SBP ↔ DBP ↔ TG ↔ LDL ↔ HDL ↔ TC
Sharma et al. (2011)	India [36]	Parallel (M/F) T2DM patients	40 (20/20)	42 μg chromium in 9 g Brewer's yeast (35–67 years)	4 weeks	↓ SBP ↔ DBP
Kleefstra et al. (2006)	Netherlands [38]	Parallel (M/F) T2DM patients	32 (15/17)	1000 μg chromium picolinate (60.5 years)	25 weeks	↔ SBP ↔ DBP
Ali et al. (2011)	USA [39]	Cross-over (M/F) MetS with IGT	60	500 μg chromium picolinate (56.9 years)	25 weeks	↔ SBP ↔ DBP
Nussbaumerov et al. (2018)	Czech Republic [40]	Parallel (M/F) MetS with IGT	65 (33/32)	300 μg chromium- enriched (57.5 years)	24 weeks	↔ SBP ↔ DBP ↔ TG ↔ LDL ↔ HDL ↔ TC
Kalbasi et al. (2013)	Iran [41]	Parallel (M/F) T2DM patients	60 (30/30)	200 μg chromium- enriched (Not reported)	12 weeks	↔ SBP ↔ DBP
Farrokhian et al. (2019)	Iran [34]	Parallel (M/F) T2DM patients	64 (32/32)	200 μg chromium picolinate (59.4 years)	12 weeks	↔ SBP ↓ DBP ↔ LDL ↔ HDL ↔ TC ↔V LDL
Stein et al. (2013)	USA [42]	Parallel (M/F) HIV patients	39 (20/19)	1000 μg chromium picolinate (47.4 years)	8 weeks	↔ SBP ↔ DBP
Imanparast et al. (2019)	Iran [43]	Parallel (M/F) T2DM patients	92 (23/23/23/23)	500 μg chromium picolinate (51 years)	17 weeks	↔ SBP ↔ DBP ↔ TG ↔ LDL ↔ HDL ↔ TC
Chen et al. (2013)	Taiwan [44]	Parallel (M/F) T2DM patients	66 (38/28)	400 μg chromium (53.7 years)	16 weeks	↔ SBP ↔ DBP
Vrtovec et al. (2005)	Slovenia [45]	Cross-over (M/F) T2DM patients	50	1000 μg chromium picolinate (Not reported)	13 weeks	↔ SBP ↔ DBP ↔ TC
Uusitupa et al. (1983)	Finland [66]	Cross-over (M/F) T2DM patients	20	200 μg trivalent (37–68 years)	6 weeks	↔ TC ↔ TG ↔ HDL ↔ LDL
Rabinowitz et al. (1983)	USA [110]	Cross-over (M) T2DM patients	56	200 μg (52–58 yeras)	16 weeks	↔ TC ↔ TG
Hunt et al. (1985)	USA [111]	Parallel (M/F) Diabetic & non-diabetic subjects	39 (22/17)	272 μg chromium yeast (50–74 yeras)	12 weeks	↔ TC ↔ TG ↔ HDL
Abraham et al. (1992)	Israel [65]	Parallel (M/F) atherosclerotic patients	25 (13/12)	250 μg chromium chloride (63.6 years)	12 weeks	↓ TG ↓ VLDL ↑ HDL ↔ TC ↔ LDL
Bahijiri et al. (2000)	Saudi Arabia [59]	Cross-over (M/F) T2DM patients	78	200 μg chromium (36–68 years)	8 weeks	↓ TG ↑ HDL
Ghosh et al. (2002)	India [68]	Cross-over (M/F) T2DM patients and healthy subjects	50	400 μg chromium picolinate (53.5)	12 weeks	↔ TG ↔ LDL ↔ HDL ↔ TC
Iqbal et al. (2009)	USA [69]	Parallel (M/F) Obese non-diabetic patients	60 (30/30)	1000 μg chromium picolinate (47.7 years)	16 weeks	↔ TG ↔ LDL ↔ HDL ↔ TC
Racek et al. (2006)	Denmark [99]	Parallel (M/F) Diabetic subjects	36 (19/17)	400 μg chromium as enriched yeast (61.3 years)	12 weeks	↔ TG ↔ LDL ↔ HDL ↔ TC
Król et al. (2011)	Poland [112]	Cross-over (M/F) T2DM patients	20	500 μg chromium (37–63 years)	8 weeks	↔ TG ↔ LDL ↔ HDL ↔ TC
Guimaraes et al. (2013)	Brazil [64]	Parallel (M/F) Overweight diabetic subjects	42 (16/13/13)	50 μg and 200 μg of chromium nicotinate (50.6 years)	12 weeks	↔ TC ↔ LDL ↓ TG ↑ HDL
Parsaeyan et al. (2013)	Iran [60]	Parallel (M/F) Diabetic subjects	93 (43/50)	200 μg chromium picolinate (52.9 years)	12 weeks	↓ TC ↓ LDL ↓ TG ↑ HDL
Tavakoli-Talab et al. (2020)	Iran [61]	Parallel (M/F) Diabetic subjects	41 (22/19)	400 μg chromium picolinate (50.8 years)	8 weeks	↓ TC ↓ LDL ↔ TG ↔ HDL

***Abbreviations****: M: Male. F: Female; TG: Triglyceride; BP: Blood Pressure; SBP: Systolic Blood Pressure; IGT:Iimpaired glucose tolerance; DPB: Diastolic Blood Pressure; T2DM: Type 2 diabetes mellitus; HDL: High Density Lipoprotein; LDL: Low Density Lipoprotein; VLDL: Very Low Density Lipoprotein TC: Total Cholesterol; MetS: Metabolic syndrome; ↓:****Decrease; ↑: Increase; ↔: No effect***.

These conflicting findings might be probably due to several reasons including small sample size, an insufficient dose of Chromium, short duration of intervention, a combination of Chromium with other substances, and various forms of Chromium such as chromium chloride, chromium nicotinate, chromium picolinate, and chromium yeast [47]. Despite above-mentioned reasons, the Chromium functional mechanism involved in blood pressure is not still clear. Although animal studies revealed the possible mechanisms of the effect of Chromium supplementation on blood pressure due to boosting insulin action and its effects on improving lipid profile [48]. Also it has been shown that Chromium consumption can improve blood pressure in hypertensive subjects which may be related to lower renin-angiotensin system activity, reduced angiotensin-converting enzyme activity, and increased NO system activity [[49], [50], [51]]; (Fig. 1). Future mechanistic investigations are needed to reveal the possible mechanism of the effects of Chromium on blood pressure.

**Fig. 1:** The probable anti-hypertensive and lipid profile lowering effects of Chromium **Abbreviations**. RAAS, Renin-Angiotensin-Aldosterone System; PPARs-ϒ, Peroxisome proliferator-activated receptors-ϒ; LDL, Low density lipoprotein; TG, Triglyceride.

### 1.2 Chromium effects on lipid profile

T2DM is the most costly chronic disease worldwide. There is a strong correlation between global *deaths* due to *diabetes* and CVDs [52]. In diabetic individuals, the probability of heart attack along with other health conditions like hypertension, dyslipidemia, and obesity, is higher than the normal subjects [53]. There is a strong correlation between obesity and visceral adiposity with CVDs, insulin resistance and diabetes [[54], [55], [56]]. It should be mentioned that insulin resistance is suggested to be associated with metabolic syndrome, a cluster risk factors related to classic CAD such as hypertension, lipid abnormalities and impaired glucose tolerance. Several studies refer to the role of oxidative stress in insulin resistance and its link with visceral adiposity [55]. Hence, the main ways to prevent these conditions are dietary and lifestyle changes. One of the main risk factors of CVDs is dyslipidemia, which its prevalence is considerably high in CVD patients [57]. These patients generally experience abnormal lipid and lipoprotein levels including high levels of cholesterol (hypercholesterolemia), triglycerides (hypertriglyceridemia), and low-density lipoprotein-pattern. They are also suggested to apply the dyslipidemia therapy via single nutrients like minerals and vitamins [58].

Several studies worked on the effect of Chromium supplementation on lipid profile during different periods of intake. Based on the results of those studies, Chromium intake plays a positive role in ameliorating T2DM risk factors and lipid profile [41,42,[59], [60], [61]]. It is worth mentioning that Chromium supplementation is termed as ‘glucose tolerance factor’ since it is a significant mediator involved in regulating the glucose and lipid metabolism [62]. This supplementation aids the reduction of body weight as well as improves the blood lipid profile, therefore it is a well-known supplement applied for body weight loss [63]. Guimaraes et al. reported that T2DM patients during 12 weeks with 50 μg and 200 μg of Chromium nicotinate intake showed increased serum HDL and lower triglycerides, even though no change in serum cholesterol or blood glucose [64]. The same result has been reported in atherosclerotic patients that 250 μg Chromium chloride during 12-week could decrease the triglyceride and very low-density lipoprotein (VLDL) levels [65]. However, in other studies, no changes were reported in lipid profiles [38,39,43,[66], [67], [68], [69]]. In Nussbaumerova et al. study Chromium-enriched yeast (200 μg of elementary Chromium in the morning and the amount of 100 μg in the evening) in 70 patients suffered from metabolic syndrome and impaired glucose tolerance (IGT) has no significant alteration in lipid parameters [40]. In line with this result, another investigation on metabolic status in diabetic patients with CHD revealed no change in lipid profile after 12-week supplementation of 200 μg Chromium [34], [Table 1], In one meta-analysis study conducted in 2022, Zhao et al. showed that supplementation in patients with diabetes improved glycosylated hemoglobin, but its effects on blood lipid levels were not significant [70]. These contradictory results are probably due to the low dose of chromium supplementation as well as the health conditions of the participants.

Several possible mechanisms of the Chromium effect on the lipid profile have been proposed. The main molecular mechanism related to Chromium is the increased expression of several genes. These genes include low-density lipoprotein receptor (LDLR), peroxisome proliferator-activated receptors-ϒ (PPARs-ϒ) and Glucose transporter (GLUT) 1,3 and 4 [71]. One possibility is that the overexpression of PPAR- ϒ may lead to improve the insulin sensitivity and lipid profile and reduce the insulin resistance [72,73]. Of note, PPAR- ϒ is proposed as an essential regulator of glucose, lipid and insulin which is widely expressed in different tissues of the body [74]. Moreover, the major glucose transporter protein which regulates the glucose uptake is GLUT 4. The concentration of insulin can affect the expression of GLUT 4 [75]. Besides, GLUT 1 and 3 play a role in regulation of blood glucose and lipid homeostasis [76]. It has been proposed that over-expression of the aforementioned proteins may be caused from increased serum insulin levels by using Chromium supplementation. With respect to lipid metabolism, LDL receptors are considered as an important regulator of cholesterol metabolism [77]. It also seems that Chromium can reduce lipogenesis and improve lipid profile by influencing the expression of the sterol regulatory element-binding protein 1 (SREBP-1) gene [78]. It can be concluded that Chromium supplementation may be a practical treatment to control the lipid profiles while reducing drug dosage in T2DM. Of note, it is obvious that a larger scale of investigations should be performed to find the convenient chemical forms of chromium, the effective time, and the exact dosage required to achieve optimal responses in patients.

### 1.3 Chromium effects on inflammatory indices

Inflammatory indices are considered to increase the risk of mortality from CVDs in general populations [79]. These markers are proposed to be novel risk factors that can be utilized for CVDs prediction [79]. Numerous studies showed that Chromium supplementation could play a crucial role in inflammation and immune activation [80]. In previous studies, Chromium supplementation was introduced to inhibit the inflammation indices in humans and animals [35,81,82]. In addition, Zhang et al. in their meta-analysis revealed the inverse association between Chromium supplementation and the level of inflammatory biomarkers including hs-CRP, tumor necrosis factor-α (TNF-α), and interleukin-6 (IL-6), as main risk factors of CVDs [83]. TNF-α is an important cytokine involved in the acute phase reaction, and dysregulation of TNF-α might be associated with heart diseases like atherosclerosis [84]. IL-6 is another factor mediating the acute phase response, this cytokine is involved in many processes such as inflammation, host defense, cancer, metabolic regulation, cellular growth, some neural functions, and hypertrophy. The level of IL-6 in plasma has been correlated with blood pressure, plasma angiotensin II levels, and vascular hypertrophy [85]. In a study by Farrokhian et al. the effects of Chromium administration on inflammation biomarkers among diabetic patients with CHD were investigated, after the 12-week intervention with the intake of 200 μg chromium picolinate, a significant decrease in serum hs-CRP was reported which was comparable with placebo [34]. Likewise, Amiri Siavashani et al. showed that the Chromium supplementation (200 μg/day) could lead to decrease in hs-CRP level as well as IL-1 downregulation without change in the expression level of IL-8 and TNF-α in women with polycystic ovary syndrome (PCOS) after 8 weeks intervention [86]. In line with this finding, Jamilian et al. reported a reduction of hs-CRP after 8 weeks of intake of 200 μg chromium supplements in PCOS patients [87]. However, in several investigations Chromium supplementations had no effect on the hs-CRP level [35,40,69]. These disputing results may be due to several reasons including using the heterogeneous and small patient population, cooperation of a single center to perform studies, short duration of chromium application, the different levels of chromium deficiency in individuals, and the inadequate amount of chromium which was applied in studies. In four studies, Chromium intake did not affect the levels of TNF-α in patients [35,44,88,89]. For example, in Yanni et al. the study, this contradictory result was proposed to be owing to the short duration of intervention, climate condition during the study, and the small number of participants and their diets [35]. In addition, Saiyed et al. suggested that the main limitation in their study was the lack of sufficiently powered for stratification based on medication usage, which may lead to this debating result [89]. Nevertheless, Imanparast et al. reported a reduction of TNF-α level in T2DM patients after 28 weeks of intervention of 500 μg chromium picolinate alongside with vitamin D3 at a dosage of 50000 IU/week [43]. The decreased level of TNF-α in this investigation might be due to the co-supplementation of chromium and vitamin D3 with an anti-inflammatory properties [90]. Furthermore, in the aforementioned study, the duration of intervention was 28 weeks, which was longer compared to other studies. With respect to IL levels after Chromium consumption, in a study by Jian et al. the level of IL-6 and IL-8 did not change after 12 weeks of intervention with 400 μg chromium picolinate/day [88], even though in another investigation by Chen et al. a decrease in IL-6 level was reported during a 16-week intervention with 200 μg/day chromium chloride, although this intervention did not have a significant effect on TNF-α level [44]. The reason for this difference in the results of two studies might be due to the type of applied supplement and the duration of the intervention.

It is worth mentioning that Chromium supplementation acts as an anti-inflammatory and anti-oxidative agent which inhibits nuclear factor kappa B (NF-κB) activation [34]. In detail, Chromium leads to increased activity of the cellular energy sensor 5’ AMP‐activated protein kinase (AMPK) [78]. Thus, AMPK activation results in deacetylation of NF‐κB and inhibits NF‐κB signaling and expression of cytokine [91]. Hence, Chromium supplementation may have beneficial effects on patients with T2DM and CVDs. Moreover, this supplement may be potential as an adjunct therapy for subjects with two mentioned diseases.

### 1.4 Chromium effects on oxidative stress markers

Elevated oxidative stress has been considered as a potential cause of CVDs [92]. It has been proven that the cells need to have a proper balance between the presence of reactive oxygen species (ROS) and antioxidants for normal function [93]. In contrast, elevated level of ROS results in damage to cellular macromolecules including DNA, lipids, and proteins, ultimately contributing to necrosis and apoptosis [94]. The result of increased ROS would be decreased availability of NO and vasoconstriction, leading to arterial hypertension. It has been indicated that ROS has a negative impact on myocardial calcium handling, causing arrhythmia, and augments cardiac remodeling through the induction of hypertrophic signaling and apoptosis [92] Eventually, ROS has also been revealed as a major factor to promote atherosclerotic plaque formation [92].

Previous studies indicated that Chromium supplementation potentially has an antioxidant effect [95] Some conditions like diabetes and chronic hyperglycemia were linked with an increase in oxidative stress, that may leading to CVDs [96]. It has been proven that oxidative stress levels are positively related to an increase in insulin resistance and inflammation. For instance, Lai et al. examined the effect of chromium supplementation on oxidative stress indices in T2DM patients. After 24 weeks of Chromium-enriched yeast administration at a dose of 1000 μg once per day (chromium-enriched Yeast alone or in combination with Vitamin E & C), the level of *glutathione peroxidase (GPx)* significantly elevated in the recipients of Chromium [97]. Besides, The results of the systematic review and meta-analysis study by Morvaridzadeh et al. revealed that supplementation with Chromium causes a significant improvement in the levels of factors related to oxidative stress, such as an increase in glutathione (GSH) and total antioxidant capacity (TAC) and decrease in *malondialdehyde* (MDA) levels [98].

On the contrary, several investigations revealed that there is no association between chromium administration and change in activities or levels of antioxidant enzymes in the group receiving Chromium. In this regard, Nussbaumerova et al. indicated that the use of 300 μg Chromium in the form of Chromium-enriched yeast in 70 patients with T2DMs after 24 weeks, did not show a significant elevation in the antioxidant enzyme levels (plasma *glutathione* peroxidase (GSH-Px) and GSH) [40]. In addition, Anderson et al. demonstrated that oral supplementation of 400 μg/d Chromium picolinate alone or in combination with zinc for 6 months did not alter the activity of antioxidant enzymes including superoxide dismutases (SODs) and GPx [95]. In another study conducted by Racek et al. they revealed that administration of 400 μg/d Chromium-enriched yeast in T2DMs after 12 weeks did not lead to a significant alteration in the levels of GSH, GSH-px, and SOD [99]. Moreover, Cheng et al. reported that daily application of 1000 μg Chromium picolinate supplementation (as chromium yeast) did not affect the antioxidant enzyme activities like SOD, GPx, and catalase (CAT) in T2DMs after 6 months [44]. In another investigation by Yanni et al. the supplementation of Chromium-enriched yeast compared to the whole wheat bread (WWCrB) group, showed a non-significant change in total antioxidant capacity after 12 weeks of intervention [35]. These conflicting results in the aforementioned studies might stem from the different duration of chromium intervention, application of Chromium in combination with yeast, zinc, or Vitamin E & C (Table 2).

**Table 2:** Effects of chromium supplementation on inflammatory and oxidative stress markers in clinical trial studies.

Author (year)	Country (Reference number)	Study design (Sex) Heath Situation	Participants numbers (Intervention/Placebo)	Dose of chromium Administered/day (Mean age)	Duration	Outcome measures
Jamilian et al. (2016)	Iran [87]	Parallel (F) PCOS patients	60 (30/30)	200 μg chromium picolinate (18–40 years)	8 weeks	↓ hs-CRP ↑ TAC ↔ GSH ↓ MDA ↔ NO
Racek et al. (2006)	Denmark [99]	Parallel (M/F) Diabetic subjects	36 (19/17)	400 μg chromium as enriched yeast (61.3 years)	12 weeks	↑ GSH ↑ GSHPx ↔ SOD ↔ MDA
Yanni et al. (2018)	Greece [35]	Parallel (M/F) T2DM patients	30 (15/15)	400 μg chromium- enriched yeast bread (65.8 years)	12 weeks	↔ CRP ↔ TAC ↔ IL-6 ↔ TNF-α
Parsaeyan et al. (2013)	Iran [60]	Parallel (M/F) Diabetic subjects	93 (43/50)	200 μg chromium picolinate (52.9 years)	12 weeks	↔ MDA
Farrokhian et al. (2019)	Iran [34]	Parallel (M/F) T2DM patients	64 (32/32)	200 μg chromium picolinate (59.4 years)	12 weeks	↓ hs-CRP ↑ TAC ↓ MDA ↑GSH
Nussbaumerov et al. (2018)	Czech Republic [40]	Parallel (M/F) MetS with IGT	65 (33/32)	300 μg chromium- enriched (57.5 years)	24 weeks	↔ hs-CRP ↔ GSH ↔ GSHPx
Amiri Siavashani et al. (2018)	Iran [86]	Parallel (F) PCOS patients	40 (20/20)	200 μg chromium picolinate (33.8 years)	8 weeks	↓ hs-CRP ↔ NO
Iqbal et al. (2009)	USA [69]	Parallel (M/F) Obese non-diabetic patients	60 (30/30)	1000 μg chromium picolinate (47.7 years)	16 weeks	↔ hs-CRP ↔ Urinary isoprostanes
Chen et al. (2014)	Taiwan [44]	Parallel (M/F) T2DM patients	66 (38/28)	200 μg chromium chloride (53.3 years)	16 weeks	↓ IL-6 ↔ TNF-α
Imanparast et al. (2019)	Iran [43]	Parallel (M/F) T2DM patients	92 (23/23/23/23)	500 μg chromium picolinate + vitamin D3 at a dosage of 50000 IU/week	28 weeks	↓ TNF-α
Jian et al. (2012)	USA [88]	Parallel (M/F) T2DM patients	74 (25/25/24)	400 μg chromium picolinate (51.1 years)	12 weeks	↔ TNF-α ↔ IL-6 ↔ IL-8
Saiyed et al. (2016)	USA [89]	Parallel (M/F) T2DM patients	25 (12/13)	400 μg chromium picolinate (50.7 years)	12 weeks	↔ TNF-α
Anderson et al. (2001)	Tunisia [95]	Parallel (M/F) T2DM patients	110 (27/27/27/29)	400 μg chromium picolinate alone or in combination with zinc (53.6 years)	24 weeks	↔ GPx ↓ TBARS
Cheng et al. (2004)	Taiwan [113]	Parallel (M/F) T2DM patients	68 (34/34)	1000 μg chromium picolinate (51.6 years)	24 weeks	↓ TBARS ↑ TAS ↔ SOD ↔ GPx ↔ Catalase
Kooshki et al. (2020)	Iran [114]	Parallel (M/F) NAFLD patients	46 (23/23)	400 μg chromium picolinate (20–65 years)	12 weeks	↑ TAC ↓ MDA ↔ GPx ↑ SOD
Lai et al. (2008)	Taiwan [97]	Parallel (M/F) T2DM patients	30 (10/10/10)	1000 μg chromium- enriched Yeast alone or in combination with Vitamin E & C (51.7 years)	24 weeks	↓ TBARS ↑ TAS ↔ SOD ↑ GPx ↔ Catalase

***Abbreviations****: M: Male. F: Female; GSH: Glutathione; GSHPx: Glutathione peroxidase; SOD: Superoxide dismutase; MDA: Malondialdehyde; PCOS: Polycystic Ovary Syndrome; T2DM: Type 2 diabetes mellitus; TBARS: Thiobarbituric acid reactive substances; CRP: C-Reactive Protein; NO:Nitric oxide;* TAS*: Total antioxidant status; ET-1; Endothelin-1; IL-1β: Interleukin 1 beta; TNF-α: Tumor necrosis factor alpha; GSH: Glutathione; GPx: Glutathione peroxidase; SOD:* Superoxide dismutase*; NAFLD: Non-alcoholics fatty liver patients; MDA: Malondialdehyde; TAC: Total antioxidant capacity; ↓:****Decrease; ↑: Increase; ↔: No effect***.

Chromium supplementation plays a critical role in improving oxidative stress by diminish circulating levels of lipid peroxidation level [100]. Despite the fact that the possible mechanism for improving MDA levels by Chromium supplementation is unclear, animal studies showed that Chromium supplementation leads to reduction of MDA and may be associated with its antioxidant features [101,102]. Of note, MDA-lowering effects after Chromium consumption might be associated with the inhibition of epinephrine owing to the Chromium insulinotropic effect [103]. Besides, this supplementation noticeably improves antioxidant enzymes’ activity and increases the levels of antioxidant indices in both human and animal investigations [100].

The ROS produced by mitochondria could be neutralized by SODs, CAT, GPx, glutathione reductase (GR), glutathione S-transferases (GSTs) [100]. Chromium generally decrease oxidative stress via various ways such as diminish ROS production, scavenging ROS, and interfering with ROS activity [40], or through the activation of GR or some other enzymes involved in detoxification of ROS and nitrogen species, leading to elevated activities of SOD, CAT, GPX, GR, and GSTs enzymes. The result can be improved levels of GSH and total antioxidant capacity (TAC) [100,104]. It should be mentioned that nicotinamide adenine dinucleotide phosphate (NADPH) as an essential electron donor, can be risen by Chromium administration, and it can be possible by increasing the activity of the glucose-6-phosphate dehydrogenase enzyme (G6PD) [105]. This process would result in changing GSSG (glutathione disulfide) into GSH (94). This supplement aids at Nrf-2 up-regulation and nuclear translocation, leading to antioxidant response element (ARE) [106]. Nrf-2 plays a key role in the expression of some antioxidant and detoxifying enzymes such as NAD (P)H: Quinone oxidoreductase 1 (NQO1), heme oxygenase-1 (HO-1), GPx, and SOD [100,107,108]. Furthermore, Chromium through expanding the level of the free radical scavenging enzymes involved in oxidative stress, contributes to reducing the interaction among hydrogen peroxide and superoxide radicals with nitric oxide [109] (Fig. 2).

**Fig. 2:** The probable anti-inflammatory and antioxidant effects of Chromium. **Abbreviations**: AMPK, AMP‐activated protein kinase; TNF-α, Tumor Necrosis Factor Alpha; CRP, C-Reactive protein; IL-6; Interleukin 6; NF-κB; nuclear factor kappa B; SODs, Superoxide dismutase; CAT, Catalase; GPX, Glutathione peroxidase; GR, Glutathione reductase; MDA, Malondialdehyde; SREBP-1, Sterol regulatory element-binding protein 1; ROS, Reactive oxygen species; GSTs, Glutathione S-transferases; NRF-2, Nuclear factor erythroid 2–related factor 2; NAD (P)H, Nicotinamide adenine dinucleotide (phosphate) dehydrogenase; NQO1, Quinone oxidoreductase 1; HO-1, Heme oxygenase-1.

## 2 Conclusion

This review article summarized that the administration of minerals and other supplements may be an accessible and safe therapy for heart diseases. Chromium supplementation is a vital mineral that plays a crucial role in the regulation of insulin action. Based on recent investigations, trivalent Chromium functions as a cofactor which increases the effects of insulin mediates the metabolism of fat, carbohydrates, and protein, and thus may plays a role in control of some risk factors of CVDs and T2DM. In this regard, Chromium can affect blood pressure, lipid profile, inflammatory indices, and oxidative stress markers. In detail, it may reduce the SBP and DBP, therefore can affect blood pressure. In addition, it can improve the lipid profile via increase the expression of several genes including PPARs-ϒ, GLUT 1,3 and 4, and LDLR. Furthermore, it might lead to lowering levels of the inflammatory indices by inhibiting NF-kB activation. Besides, it may affect and improve the oxidative stress markers through reducing ROS production, scavenging the ROS, interfering with ROS activity, and activation of enzymes involved in detoxification of ROS and nitrogen species. In order to find any potential role of Chromium supplementation in CVD conditions, further well-designed studies are required.

## Data availability statement

Data sharing is not applicable to this article as no datasets were generated or analyzed.

## Declaration of competing interest

The authors declare that they have no known competing financial interests or personal relationships that could have appeared to influence the work reported in this paper.
